The article "Analysis on Value of Applying Serum miR-144 and miR-221 Levels in Diagnosing Atherosclerosis" was retracted in 2023. Reason: concerns about the peer review.

# Analysis on Value of Applying Serum miR-144 and miR-221 Levels in Diagnosing Atherosclerosis

**DOI:** 10.1155/2022/2261854

**Published:** 2022-01-25

**Authors:** Jianxiu Zhang, Qian Cao, Zhenying Zhang, Chenguang Du, Lizhong Wang

**Affiliations:** ^1^Cardiac Rehabilitation Centre, Beijing Rehabilitation Hospital of Capital Medical University, Beijing 100144, China; ^2^Cardiac Rehabilitation Centre, College of Traditional Chinese Medicine, North China University of Technology, Tangshan, Hebei Province 063210, China

## Abstract

**Objective:**

To explore the value of serum miR-144 and miR-221 in diagnosing atherosclerosis (AS).

**Methods:**

The clinical data of 52 AS patients treated in the department of cardiovascular medicine of our hospital from August 2019 to August 2020 were retrospectively analyzed, and 53 healthy persons were selected from the physical examination center at the same period as the control group. By measuring the indicators including the serum vascular endothelial growth factor (VEGF), superoxide dismutase (SOD), miR-144, and miR-221 in patients of both groups, their value of diagnosing AS was analyzed.

**Results:**

Compared with the control group, the AS group obtained significantly higher serum miR-221 and miR-144 expression levels (*P* < 0.001), significantly higher mean serum homocysteine (Hcy) level value (*P* < 0.001), lower mean serum SOD level (*P* < 0.001), and significantly higher level values of serum VEGF, nuclear factor-kappaB (NF-kB), and transforming growth factor-*β* (TGF-*β*) (*P* < 0.001), and the area under ROC curve, sensitivity, and specificity of combining miR-221 with miR-144 were significantly higher than those of single diagnosis.

**Conclusion:**

Serum miR-221 and miR-144 expression levels are increased in AS patients, and combining the two indicators in diagnosis is more accurate and can provide an accurate basis for diagnosis and condition assessment of AS.

## 1. Introduction

Atherosclerosis (AS) is a slowly progressive cerebrovascular disease. Research and investigations have revealed that [1, 2] approximately 20 million people worldwide die from the disease each year, which is an important cause of diseases including angina, coronary heart disease, and sudden cardiac death, as well as a leading cause of death in the elderly population. Although the fatality rate of AS shows a decreasing trend with modern medical treatment technology advancing day by day, its incidence rate is still increasing. Traditionally, AS is assessed mainly by imaging methods such as ultrasound vascular examination or X-ray, but quantitative indexes of assessment are lacking. According to the research finding [3], the incidence of AS is closely related to vascular inflammation, cell proliferation and apoptosis, and lipid metabolism, which is a complex and slow process. Recently, with the intensive research on exosomes, it has been found that exosomes can act as an important medium of intercellular communication and plays a major role in the occurrence and progression of AS. Micro-RNAs (miRNAs), stably present in various body fluids as the biomarker for various types of diseases, involve in the formation of AS as the key signaling and molecular regulator (Figure 1) [4–6]. miR-144 is structurally highly conserved and involves in the occurrence and progression of cancer, and cardiovascular diseases. Foreign scholars have confirmed [7] the downregulation of miR-144 in plasma of patients with medullary carcinoma of thyroid, which in turn led to the development and progression of thyroid cancer; other studies have proved that [8] miR-144 played the role of cancer suppressor gene in cervical cancer, which provided a new direction in the later diagnosis and treatment for cardiovascular diseases. It has been proved that miR-211 is expressed abnormally in patients with epithelial ovarian cancer and closely related to the processes such as incidence, invasion, and metastasis of such disease [9, 10]. Currently, the diagnostic efficacy of miR-144 and miR-221 in AS is rarely studied, and therefore, it was analyzed herein to prevent and treat relevant cardiovascular diseases by target regulating miR-144 and miR-221 expression levels.

The article "Analysis on Value of Applying Serum miR-144 and miR-221 Levels in Diagnosing Atherosclerosis" was retracted in 2023. Reason: concerns about the peer review.

## 2. Data and Methods

### 2.1. General Information

The study was reviewed and approved by the hospital ethics committee. The clinical data of 52 AS patients treated in the department of cardiovascular medicine of our hospital (08.2019–08.2019) were selected for the retrospective study, and 52 healthy persons were screened from the physical examination center at the same period as the control group. Patients in the AS group met the diagnosis criteria of the disease, namely, abnormal blood lipid indexes and vascular stenosis lesions found in arteriography, and their clinical manifestations included angina, arrhythmia, headache, and fainting. Those with heart failure, angina, heart disease, hypertension, kidney function obstacle, and other cardiovascular diseases were excluded. Under the condition that all subjects signed the informed consent and agreed to join the study, the retrospective analysis and physical examination were conducted to all enrolled subjects, and their gender, age, BMI values, and other indicators were recorded.

### 2.2. Index Detection

#### 2.2.1. Detection of miR-221 and miR-144 Level Values

The subjects fasted for more than 10 h. Before blood drawing, relevant instruments were prepared as required. The patients took the sitting position, with an arm extended straight on the table and the tourniquet tied at the upper arm; they were instructed to repeatedly make a fist to fill the vein, a cotton stick moistened with iodophor was used to make a ring disinfection treatment at the site for venipuncture with a syringe to collect 10 ml of venous blood, blood was placed in a procoagulant containing blood collection tube, and after centrifugation at 3,500 r/min for 10 min in an intelligent high-performance centrifuge (Beckman Coulter China branch; model: Avanti JXN-30/26), the serum from the upper layer was collected for relevant index detection [11, 12].

The article "Analysis on Value of Applying Serum miR-144 and miR-221 Levels in Diagnosing Atherosclerosis" was retracted in 2023. Reason: concerns about the peer review.

The extraction of RNA in serum was conducted according to the specification of blood RNA extraction kit (Shanghai GenePharma Co., Ltd.). The extracted RNA was collected and reversely transcribed into cDNA with the genome removal reverse transcription kit (Shanghai Ruifen Biotechnology Co., Ltd.). The expression levels of serum miR-221 and miR-144 were detected by the real-time fluorescent quantitative PCR method.

#### 2.2.2. Detection of Serum Superoxide Dismutase (SOD) and Homocysteine (Hcy) Levels

The level values of serum SOD and Hcy were detected with the automatic biochemical analyzer (Shanghai Huanxi Medical Device Co., Ltd.; model: LW C200E).

#### 2.2.3. Detection of Vascular Endothelial Growth Factor (VEGF), Nuclear Factor-Kappa B (NF-kB), and Transforming Growth Factor-*β* (TGF-*β*) Levels

The cytokine levels were detected by enzyme-linked immunosorbent assay (ELISA), the VEGF and NF-kB kits were purchased from Shanghai Zhen Ke Biological Technology Co., Ltd., the FGF-*β* kits were purchased from Shanghai Win-Win Biotechnology Co., Ltd., and all operations were carried out according to the kit instructions.

### 2.3. Statistical Processing

The statistical analysis and processing of experimental data were conducted with SPSS 21.0 software, the picture drawing software was GraphPad Prism 7 (GraphPad Software, San Diego, USA), the diagnosis value was analyzed by the Mann–Whitney *U* test, and the area under receiver operating characteristic curve (ROC curve), the measurement data examined by the *t*-test and expressed by ($\bar{\text{x}}$ ± *s*), and differences were considered statistically significant at *P* < 0.05.

## 3. Results

### 3.1. Between-Group Comparison of Basic Clinical Information

Other than various blood lipid indicators, no obvious between-group differences in the gender ratio, mean age, BMI value, smoking history, and drinking history were observed (*P* < 0.05), as given in Table 1.

### 3.2. Between-Group Comparison of Serum miR-221 and miR-144 Levels

Compared with the control group, the AS group had significantly higher miR-221 expression level and significantly lower miR-144 expression level (*P* < 0.001), as shown in Figure 2.

The article "Analysis on Value of Applying Serum miR-144 and miR-221 Levels in Diagnosing Atherosclerosis" was retracted in 2023. Reason: concerns about the peer review.

### 3.3. Between-Group Comparison of Serum SOD and Hcy Level Values

Compared with the control group, the AS group presented significantly higher mean serum Hcy level values (*P* < 0.001) and significantly lower mean serum SOD level values (*P* < 0.001), as shown in Figure 3.

### 3.4. Between-Group Comparison of Serum VEGF, NF-kB, and TGF-*β* Level Values

The serum VEGF, NF-kB, and TGF-*β* level values were significantly higher in the AS group than in the control group (*P* < 0.001), as given in Table 2.

### 3.5. Diagnosis Value of Serum miR-221 and miR-144 Levels for AS

The areas under the ROC curves of serum miR-221 and miR-144 levels for the diagnosis of AS was 0.670 and 0.613, respectively, and the area under the ROC curve of combined diagnosis was 0.858 (Table 3 and Figures 4–6).

## 4. Discussion

AS will cause arterial wall thickening, vessel stenosis, and vascular elasticity decrease, which is the main pathological basis of coronary heart disease, cerebral infarction, and peripheral ischemic vascular disease [13] and chronic inflammatory disease triggered by various factors. Since the early symptoms of the disease are not obvious, most patients have entered middle and late stages when diagnosed, seriously affecting the prognosis. Intravascular ultrasound (IVUS) examination is a common method for the diagnosis of AS [14–16], but it cannot accurately obtain the internal fine structure of local plaques, has less significance for identifying their vulnerability, and is an invasive tomographic technique [17]. On people's deeper exploration of serum biology, it is found that inflammation extends through the whole occurrence and progression process of AS, a long-term formed and progressed chronic inflammatory response, while serum marker levels are relatively stable and less affected by other factors, presenting higher sensitivity and specificity. Studies have shown that multiple cell-derived exosomal miRNAs are involved in this inflammatory process [18], exacerbating the disease progression of AS by causing inflammatory responses in its targeted cells and then leading to the formation of endothelial cell insufficiency, monocyte adhesion, foam cell, and vascular remodeling in the arterial wall. Among them, miR-221 accelerates the progression of AS by participating in the inflammatory response, activating its target genes, and causing dysfunction of the vascular endothelial membrane in patients. In the study conducted by foreign scholars [19] on a rat model of inflammation caused by chronic intake of sucrose, by detecting the exosomes in rats' blood, it was found that their miR-221 expression in plasma was significantly elevated, from which it could be speculated that miR-221 in plasma exosomes might be involved in the inflammatory response. Another study also found [20] that upregulated miR-221 expression could inhibit the cell cycle regulator p27kip1 in vascular smooth muscle cells, thereby mediating vascular calcification to cause atherosclerosis and stenosis. In this study, by detecting the expression levels of serum miR-221 in AS patients and in healthy persons, it was found that the miR-221 expression level was significantly higher in AS patients (*P* < 0.001), which was proved in the study by Elbaek et al. [21].

The article "Analysis on Value of Applying Serum miR-144 and miR-221 Levels in Diagnosing Atherosclerosis" was retracted in 2023. Reason: concerns about the peer review.

As an evolutionarily highly conserved miRNA, miR-144 is mapped on chromosome 17 in humans and exists as a miR-144/miR-451 gene cluster [22]. miR-144 levels in tissues are also of a great value in the diagnosis and prognosis evaluation of malignant tumors, and its clinical utility has been demonstrated in diseases such as breast cancer, oral squamous cell cancer, and colon cancer cancer [23]. Studies have found that [24] miR-144 is highly expressed in cardiomyocytes, and its high expression level can promote myocardial oxidative stress, thereby inducing myocardial injury related diseases, and its key role in the occurrence and progression of cardiovascular diseases have been confirmed by several foreign clinical trials. In this study, it was found that the serum miR-144 expression level in AS patients was significantly higher than that in the healthy group, and Lu et al. [25] in their study found that miR-144 expression in AS plaques and vascular smooth muscle cells (VSMCs) would gradually elevate as the disease progressed, presumably due to the imbalance of methylation and demethylation systems in vivo causing increased methylation of the miR-144 promoter.

An ideal serum marker shall have high specificity and sensitivity. In this study, miR-144 was found to be under expressed in the serum of AS patients, and its area under the ROC curve for the diagnosis of AS was 0.613, whereas miR-221 had an area under the ROC curve of 0.670, which was higher than that of miR-144. But considering the low specificity of miR-144 in the diagnosis of AS, miR-221 was adopted for combined diagnosis, and as a result, the combination could improve the specificity and sensitivity of miR-144 for the diagnosis of AS, with an area under the ROC curve of 0.858. Deficiency of this study is that the small number of cases selected and the failure to consider the effect of disease type and stage on the results of the study are prone to bias of conclusions.

The article "Analysis on Value of Applying Serum miR-144 and miR-221 Levels in Diagnosing Atherosclerosis" was retracted in 2023. Reason: concerns about the peer review.

In conclusion, both miR-144 and miR-221 participate in the occurrence and progression of AS, and the combination of the two has a higher diagnosis value and can provide a new direction for the clinical diagnosis of AS.

## Figures and Tables

**Figure 1:** Effect of exosomal miRNA on AS progression.

**Figure 2:** Between-group comparison of serum miR-221 and miR-144 levels ($\bar{\text{x}}$ ± *s*). (a) The between-group comparison of miR-221 expression levels. The horizontal axis denotes the AS group and control group, and the vertical axis denotes the level. The miR-221 expression level of the AS group and control group was 10.24 ± 2.31 and 3.12 ± 0.54, respectively, and  ^*∗*^ indicates the significant between-group difference in the miR-221 expression levels (*t* = 21.841, *P* < 0.001). (b) The between-group comparison of miR-144 expression levels. The horizontal axis denotes the AS group and control group, and the vertical axis denotes the level. The miR-144 expression level of the AS group and control group was 1.31 ± 0.16 and 0.25 ± 0.07, respectively, and  ^*∗*^ ^*∗*^ indicates the significant between-group difference in the miR-144 expression levels (*t* = 44.122, *P* < 0.001).

**Figure 3:** Between-group comparison of serum SOD and Hcy level values ($\bar{\text{x}}$ ± *s*). (a) The between-group comparison of serum SOD level values. The horizontal axis denotes the AS group and control group, and the vertical axis denotes the value (*μ*g/g). The mean serum SOD level values of the AS group and control group were (477.30 ± 31.19) and (606.65 ± 32.00), respectively, and  ^*∗*^ indicates the significant between-group difference in mean serum SOD level values (*t* = 20.970, *P* < 0.001). (b) The between-group comparison of serum Hcy level values. The horizontal axis denotes the AS group and control group, and the vertical axis denotes the value (*μ*mol/L). The mean serum Hcy level values of the AS group and control group were (28.17 ± 6.20) and (9.09 ± 3.85), respectively, and  ^*∗*^ ^*∗*^ indicates the significant between-group difference in mean serum Hcy level values (*t* = 18.983, *P* < 0.001).

**Figure 4:** ROC curve of diagnosing AS with serum miR-221 expression level.

**Figure 5:** ROC curve of diagnosing AS with serum miR-144 expression level.

**Figure 6:** ROC curve of diagnosing AS with miR-221 + miR-144 expression level.

**Table 1:** Between-group comparison of basic clinical information (*n* (%), $\bar{\text{x}}$ ± *s*).

Item	AS group (*n* = 52)	Control group (*n* = 53)	*X* ^2^/*t*	*P*
Gender			0.094	0.759
Male	30 (57.69%)	29 (54.72%)		
Female	22 (42.31%)	24 (45.28%)		
Mean age ($\bar{x}$ ± *s*, years)	64.37 ± 3.26	64.42 ± 3.31	0.078	0.938
BMI ($\bar{x}$ ± *s*, kg/m^2^)	21.19 ± 1.02	21.23 ± 1.04	0.199	0.843
Smoking history	29 (55.77%)	31 (58.83%)	0.079	0.778
Drinking history	32 (61.54%)	28 (52.83%)	0.813	0.367
Total cholesterol ($\bar{x}$ ± *s*, mmol/L)	5.22 ± 0.47	3.52 ± 0.46	18.731	<0.001
Triacylglycerol ($\bar{x}$ ± *s*, mmol/L)	1.62 ± 0.46	0.84 ± 0.21	11.212	<0.001
LDL-C ($\bar{x}$ ± *s*, mmol/L)	3.56 ± 0.35	2.26 ± 0.17	24.280	<0.001
HDL-C ($\bar{x}$ ± *s*, mmol/L)	1.12 ± 0.31	1.34 ± 0.23	4.135	<0.001

The article "Analysis on Value of Applying Serum miR-144 and miR-221 Levels in Diagnosing Atherosclerosis" was retracted in 2023. Reason: concerns about the peer review.

**Table 2:** Between-group comparison of serum VEGF, NF-kB, and TGF-*β* level values ($\bar{\text{x}}$ ± *s*).

Group	*n*	VEGF (pg/ml)	NF-kB (ng/L)	TGF-*β* (ng/L)
AS group	52	432.25 ± 35.64	1.69 ± 0.36	257.83 ± 5.27
Control group	53	142.56 ± 24.26	1.04 ± 0.29	67.48 ± 4.58
*T*		48.770	10.198	197.662
*P*		<0.001	<0.001	<0.001

**Table 3:** Diagnosis value of serum miR-221 and miR-144 levels for AS.

Indicator	Area under ROC curve	Positive rate (%)	95% CI	Sensitivity (%)	Specificity (%)
miR-221	0.670	24.76	0.566–0.774	86.75	81.26
miR-144	0.613	21.90	0.505–0.721	79.25	74.27
miR-221 + miR-144	0.858	43.81	0.781–0.935	93.25	85.37

## Data Availability

The data used to support the findings of this study are available from the corresponding author upon request.

## References

[1] Gong W., Li J., Wang Y., Guangying Z. (2019). miR-221 promotes lens epithelial cells apoptosis through interacting with SIRT1 and E2F3. *Chemico-Biological Interactions*.

[2] Ni H.-Z., Liu Z., Sun L.-L. (2019). Metformin inhibits angiogenesis of endothelial progenitor cells via miR-221-mediated p27 expression and autophagy. *Future Medicinal Chemistry*.

[3] Fu Y., Li F., Zhang P. (2019). Myrothecine a modulates the proliferation of HCC cells and the maturation of dendritic cells through downregulating miR-221. *International Immunopharmacology*.

[4] Abo El Atta A. S., Ali Y. B. M., Bassyouni I. H., Talaat R. M. (2019). Upregulation of miR-221/222 expression in rheumatoid arthritis (RA) patients: correlation with disease activity. *Clinical and Experimental Medicine*.

[5] Tang X., Tu G., Yang G. (2019). Autocrine TGF-beta 1/miR-200s/miR-221/DNMT3B regulatory loop maintains CAF status to fuel breast cancer cell proliferation. *Cancer Letters*.

[6] Ravegnini G., Serrano C., Simeon V. (2019). The rs17084733 variant in the KIT 3’ UTR disrupts a miR-221/222 binding site in gastrointestinal stromal tumour: a sponge-like mechanism conferring disease susceptibility. *Epigenetics*.

[7] Feng J., Wang M., Li M. (2019). Serum miR-221-3p as a new potential biomarker for depressed mood in perioperative patients. *Brain Research*.

The article "Analysis on Value of Applying Serum miR-144 and miR-221 Levels in Diagnosing Atherosclerosis" was retracted in 2023. Reason: concerns about the peer review.

[8] Higashi Y., Mummidi S., Sukhanov S. (2019). Minocycline inhibits PDGF-BB-induced human aortic smooth muscle cell proliferation and migration by reversing miR-221-and-222-mediated RECK suppression. *Cellular Signalling*.

[9] Cheng Z., Xing D. (2019). Ginsenoside Rg3 inhibits growth and epithelial-mesenchymal transition of human oral squamous carcinoma cells by down-regulating miR-221. *European Journal of Pharmacology: International Journal*.

[10] Srinoun K., Sathirapongsasuti N., Paiboonsukwong K., Sretrirutchai S., Wongchanchailert M., Fucharoen S. (2019). miR-144 regulates oxidative stress tolerance of thalassemic erythroid cell via targeting NRF2. *Annals of Hematology*.

[11] Siddiqui M. R., Akhtar S., Shahid M., Tauseef M., McDonough K., Shanley T. P. (2019). miR-144-mediated inhibition of ROCK1 protects against LPS-induced lung endothelial hyperpermeability. *American Journal of Respiratory Cell and Molecular Biology*.

[12] Liu J., Feng L., Zhang H. (2018). Effects of miR-144 on the sensitivity of human anaplastic thyroid carcinoma cells to cisplatin by autophagy regulation. *Cancer Biology & Therapy*.

[13] Zhao M., Huang J., Gui K. (2014). The downregulation of miR-144 is associated with the growth and invasion of osteosarcoma cells through the regulation of TAGLN expression. *International Journal of Molecular Medicine*.

[14] Kalimutho M., Del Vecchio Blanco G., Di Cecilia S. (2011). Differential expression of miR-144 as a novel fecal-based diagnostic marker for colorectal cancer. *Journal of Gastroenterology*.

[15] Gao F., Wang T., Zhang Z., Wang R., Guo Y., Liu J. (2016). Regulation of activating protein-4-associated metastases of non-small cell lung cancer cells by miR-144. *Tumor Biology*.

[16] Liu F., Wang J., Fu Q. (2016). VEGF-activated miR-144 regulates autophagic survival of prostate cancer cells against Cisplatin. *Tumor Biology*.

[17] Hartley A., Haskard D., Khamis R. (2019). Oxidized LDL and anti-oxidized LDL antibodies in atherosclerosis - novel insights and future directions in diagnosis and therapy,. *Trends in Cardiovascular Medicine*.

[18] Eikelboom J. W., Connolly S. J., Bosch J. (2019). Bleeding and new cancer diagnosis in patients with atherosclerosis. *Circulation*.

[19] Zhang Y., Zhang C., Li H., Hou J. (2019). The presence of high levels of circulating trimethylamine N-oxide exacerbates central and peripheral inflammation and inflammatory hyperalgesia in rats following carrageenan injection. *Inflammation*.

[20] Van De Pol V., Vos M., Deruiter M. C., Goumans M. J., De Vries C. J. M., Kurakula K. (2020). LIM-only protein FHL2 attenuates inflammation in vascular smooth muscle cells through inhibition of the NF*κ*B pathway. *Vascular Pharmacology*.

The article "Analysis on Value of Applying Serum miR-144 and miR-221 Levels in Diagnosing Atherosclerosis" was retracted in 2023. Reason: concerns about the peer review.

[21] Mette Vestergaard E., Anders Lindholm S., Hasselbalch H. C. (2019). Cardiovascular disease in chronic myelomonocytic leukemia: do monocytosis and chronic inflammation predispose to accelerated atherosclerosis?. *Annals of Hematology*.

[22] Yu M., Niu Y., Zhou D. (2019). Hyaluronic acid-functionalized gadolinium doped iron oxide nanoparticles for atherosclerosis-targeted Mr imaging. *Journal of Biomedical Nanotechnology*.

[23] Sheng S., Xie L., Wu Y., Ding M, Zhang T, Wang X (2019). MiR-144 inhibits growth and metastasis in colon cancer by down-regulating SMAD4. *Bioscience Reports*.

[24] Kohlman-Trigoboff D. (2019). Update: diagnosis and management of peripheral arterial disease. *The Journal for Nurse Practitioners*.

[25] Lu M., Yuan S., Li S., Li L., Liu M., Wan S. (2019). The exosome-derived biomarker in atherosclerosis and its clinical application. *Journal of Cardiovascular Translational Research*.

